# Assessment of Bacteriological Quality and Physiochemical Parameters of Domestic Water Sources in Jenin Governorate: A Case Study

**DOI:** 10.1155/2023/8000728

**Published:** 2023-07-11

**Authors:** Issam A. Al-Khatib, Maher Al-Jabari, Mahmoud Al-Oqaili

**Affiliations:** ^1^Institute of Environmental and Water Studies, Birzeit University, Birzeit, State of Palestine; ^2^Mechanical Engineering Department, Faculty of Engineering and Technology, Palestine Polytechnic University, Hebron, West Bank, State of Palestine; ^3^Universal Institute of Applied and Health Research, Nablus, State of Palestine

## Abstract

Water quality of drinking water is a concern in Palestine due to possible pollution sources. There is a demand for investigating the quality of municipal water supply. This study aimed to assess the quality of domestic water in Jenin Governorate located in the north of the West Bank. The methodology of this research was based on field sampling and laboratory standard testing. The tested parameters included (1) physicochemical parameters of electrical conductivity, turbidity, total hardness, salinity, pH, and total alkalinity, (2) chemical contents including the contents of nitrate, nitrite, sulfate, chloride, sodium, potassium, aluminum, and fluoride, and (3) biological contents including total coliforms and fecal coliforms. The water quality parameters were compared with the acceptable limits set by local and international standards. The findings confirm that most of the values of the investigated parameters are within the acceptable standard limits. No pollution of heavy metals is detectable. On the other hand, there are limited pollution contents in terms of the total dissolved solid (TDS), total hardness, and calcium. Furthermore, the biological parameters indicate that there are low to very high risks in a fraction of the water quality samples in terms of total coliforms and fecal coliforms. This is believed to be due to the presence of septic tanks in the neighborhoods of the sampling locations. For these cases, biological disinfection treatments are recommended before human use with an essential need for the construction of urban sewer systems. Furthermore, water treatment for harness removal may be required.

## 1. Introduction

Water is a key component in human life either straight forwardly as drinking water or in a roundabout way as a constituent of food and is served in different utilizations in our everyday life [1–6]. Furthermore, water is an essential parameter in the public health due to possible transmission diseases [7]. The evaluation of water quality is an essential issue, and the security of water quantity is a critical point in the governmental plans and strategies [8]. Drinking water as well as entertainment and the natural life environment can be seriously influenced by contaminations [9, 10]. Chemical spills can intimidate water quality and human health.

Palestine and other countries in the Middle East suffer from water shortage due to predominantly semiarid to arid climatic conditions [11]. Water is a critical issue in the Middle East [12]. Water resources in Palestine are limited; hence, water shortage and water quality are imminent [13, 14]. There are three groundwater aquifer bowls in Palestine, which are situated in the West Bank, but controlled by Israel. An obvious lack of fresh water for domestic, industrial, and agricultural purposes was identified as one of the main issues in Palestine [15]. For example, the allowed daily consumption of water per capita in Hebron and Nablus cities in the West Bank of Palestine is nearly 50 L/day and the average daily consumption in the whole of the West Bank is 66 L/day [12, 16]. On the other hand, the WHO has set the minimum per capita daily consumption of 100 L/day [17]. Arid and semiarid areas suffer from scarcity of water resources, so the protection of existing resources is a priority for people. Water pollution occurs in the form of altering the composition of the watercourse components due to human activity, and then, the resulting water becomes less suitable for natural uses [18–23]. In the Gaza strip, a study of the quality of drinking water revealed low pH and TDS levels, while microbiological analyses showed that the total coliform for distribution points was 58 CFU/100 ml, and in the household storage tanks, it was found to be 171 CFU/100 [24]. The reduction in water quality locally and worldwide is considered one of the environmental challenges that requires urgent action [25, 26]. In fact, the decline in water quality is a reflection of poverty. Water quality is dependent on the logistics and practices of waste disposal and wastewater discharge [18, 27–31]. Municipal wastewater and waste are two of the pollution sources of water resources. The main problem of solid waste is the leaching of possible hazardous substances, the severity of which is dependent on horizontal distance to the water sources, temperature of the area, pollution content, and age [32]. The possible reasons for water pollution in the West Bank were identified to include the absence of sewage networks in many rural areas, the utilization of cesspits for domestic wastewater, and the inappropriate waste management [13]. Any released toxins can migrate into ground water resources where poisons interface with nature. Then, the ground water resources experience physical and substance changes, and they are consolidated into the earth resulting in changes in water quality [33–35]. In general, monitoring discharges of wastewater treatment plants (WWTPs) has many benefits for the protection of drinking water resources [36]. Chemical contaminations include nitrate content that may result from biological waste from humans and animals, plant debris, and seepage [37, 38]. Groundwater contamination with heavy metals, together with the geogenic presence of some toxic metals (e.g., arsenic and fluoride), is of increasing concern due to their severe ecological and public health impacts [39–41]. The main sources of heavy metal pollution are agricultural runoffs and uncontrolled discharges of wastewater from industries, including metal electroplating and mining [42]. Traffic is also an important source of heavy metal pollution [11, 43–45].

The pollution of water resources affects the quality of the municipal water supply. In addition, for municipal water supply, colored water may be obtained due to the deposited salts in the inner surface of network pipes. In the presence of manganese (Mn), there is a strong possibility for the formation of discoloration such as “black water.” According to the United States Environmental Protection Agency, the limit value of manganese is 50 *μ*g/L [46]. These pollutants in drinking water have various impacts on public health: Water hardness can cause kidney stone formation [47]. Water for human use must be free of microbiological contaminations that are pathogenic to humans [48, 49]. Water contamination with bacteria, protozoa, and viruses causes diarrhea, which can cause the death of infants (for example, cholera and hepatitis) [50, 51]. According to the World Health Organization (WHO), the diarrheal diseases globally were estimated at 3% in 2016 [40]. For noncleaned supplies, up to 10 fecal coliforms (FC) per 100 mL are permitted [52]. Sulfate content may have a laxative effect on humans, so the maximum contaminate level is 250 mg/L. Chloride concentrations above 250 ppm could affect the taste of drinking water [53]. Aluminum can lead to Alzheimer's disease [54]. The nitrate limit according to the WHO guidelines is 50 mg/L as NO_3_ [55]. On the other hand, contamination with nitrite is more dangerous as a high concentration of nitrate can lead to methemoglobinemia [56]. High concentrations of salinity cause cholera, while small quantities of salt are essential for organizing the fluid balance of the human body [57]. The ammonia limit in groundwater according to the WHO [58] guidelines is 0.2 mg/L.

Water quality is usually monitored by measuring various parameters covering chemical, physical, and microbiological characteristics [59–61]. The physicochemical parameters include total solids (TS), total dissolved solids (TDS), total suspended solids (TSS), pH, dissolved oxygen, hardness, and chlorine and sodium contents [62]. High water turbidity may reflect the pollution of water from leaching of organic matters as well as domestic and industrial wastes. High electrical conductivity (EC) reflects a high concentration of soluble salts which makes water conductive for electric current [63]. Total hardness (mg/l) is the sum of calcium and magnesium hardness. The microbial parameters include total coliforms and fecal coliforms [15, 47, 64].

Little effort was made for assessing water quality in the West Bank areas [65, 66]. In a previous case study [66], the quality of drinking water obtained from local springs in the West Bank was evaluated. The previous study assisted in promoting the public use of the springs as a water supply. The publication of such case studies responds to a need for paving the road for performing similar case studies for other regions. This appears very obviously in the high citations of the previous case study [66] within a short time period from its publication date. There are concerns about the possible contaminations of municipal water supply that require the attention of the various authorities. The Ministry of Health is interested in assessing the quality of municipal water to prevent any potential impacts on human and public health. There is a knowledge gap in the published work on chemical, physical, and biological parameters for municipal water supplies. Currently, an ongoing international research project is concerned with the quality of water in schools for promoting public health. Consequently, perfuming case studies on the quality of municipal water supply can assist the authorities (water and health) in their planning and management efforts. Furthermore, the novelty of such a case study is concentrated in providing new information with more investigated parameters for better assessment of the water quality and providing a model approach for subsequent studies in other areas (generalization). Responding to these needs, the main research objectives are measuring the chemical, physical, and biological parameters for municipal water supply in the defined research area (Jenin district), as a case study, and evaluating the suitability of water quality for human use by comparing the measured parameters with the limits set by both national and international quality standards (the Palestinian standards (PSI) and the guidelines of the WHO). The research variables included pH, EC, total hardness, concentrations of nitrate, sodium ions, total chlorine, residual chlorine, turbidity, and total and fecal coliforms.

## 2. Methodology

### 2.1. Description of the Study Area

The domain of this study was Jenin Governorate located in the north of the West Bank. It is one of the 16 governorates of the Palestinian authority. The Jenin Governorate area comprises about 10.5% of the West Bank area and is considered one of the best agricultural areas in Palestine. Most of municipal administration of this governorate land is under the Palestinian authority. It is bordered by Nablus from the south and by Tulkarem from the southwest. Its location is between 90 and 750 m above sea level, and the highest elevation is at Jabal Hureish, while the lowest elevation is at El Mukhabba area [67]. Jenin Governorate is located above the Northeastern Groundwater Basins, the capacity of which is about 140 MCM/year [68]. Groundwater can be obtained at 50 m below the ground surface. The other sources of water include seasonal lakes such as Marj Sanur. The daily water consumption per capita in Jenin Governorate is about 50.2 L/day [69]. The projected mid-year population for Jenin Governorate in 2022 is 345875 persons [70].

### 2.2. Sampling

The sampling was performed during 2018 and 2019 from villages, towns, and cities in Jenin district in the West Bank of Palestine. The samples of drinking water were taken from wells, houses, restaurants, and others. The samples were collected by the Palestinian Ministry of Health to ensure the chemical, physical, and biological qualities of the drinking water. The samples were collected in pyrex-sterilized glass bottles (1000 mL), filtered through a 0.45 *µ*m filter (Schleicher and Schuell ME 25, Taufkirchen, Germany), divided into two fractions, and stored at 4°C. Tables 1–3 list the distribution of samples based on the investigated parameters.

### 2.3. Analysis

Water samples were taken by field crew and were then transferred to the Palestinian public health laboratories where each parameter was analyzed. The physicochemical, chemical, and biological characteristics were measured according to the standard testing procedures. The tools used included a portable digital pH meter, an EC meter, a turbidity meter, inductively coupled plasma mass spectrometry (ICP-MS), and membrane filtration. The water samples taken for analyses of cations and trace metals were acidified (pH < 1.5) with analytical grade concentrated nitric acid.

The pH and conductivity were measured in the field immediately after or during sampling, using a portable HACHsensION1 multimeter, with a combined electrode, and a portable HACH conductivity meter (HACH, Loveland, CO, USA). The total dissolved solid (TDS) and the salinity were measured using a salinity meter, Hach CO150 (Hach Company, Loveland, Columbia, USA). The remaining physicochemical parameters were tested using a DR 2400 spectrophotometer as demonstrated elsewhere [71]. The concentrations of Ca, Mg, Al, Fe, K, Na, and Ag were analyzed using ICP-MS (Agilent Technologies 7500 Series, Agilent, Santa Clara, CA, USA). The total and fecal coliforms counts were measured by the membrane filtration technique [72]. The measured parameters for each of the collected samples were tabulated, and then, the mean values and standard deviations were estimated and compared with the limits set by the WHO and the PSI.

## 3. Results and Discussion

### 3.1. Physiochemical Parameters

The results of the physiochemical parameters of the drinking water in Jenin Governorate along with allowable limits of the PSI [73] standards and the WHO [58] guideline values are listed in Table 4. Table 4 lists the range, the mean, and the standard deviation for each measured physiochemical parameter.

The values of electrical conductivity are within the range of 242–1833 *μ*S/cm, and the mean value is 890 ± 302 *μ*S/cm.  Table 5 lists the classifications of water quality for various ranges of EC and the percentage of samples in each range. All measured values of EC were within the acceptable limit set by the WHO and PSI standards (2000 *μ*Scm^−1^): the majority of the tested samples (77%) were classified as permissible, while 19.2% were classified as good and 3.8% were classified as excellent. Overall, 100% of the samples are within the PSI and WHO standards, and hence, there are no concerns regarding the soluble salts. The observed wide range of EC is an indication of the content of dissolved salts such as sodium chloride and potassium chloride. The values of the salinity are within the range of 0.01–0.050%, and the average value is 0.07 ± 0.10%. High concentrations of salinity lead to diarrhea and water-borne diseases such as cholera. Salinity is related to electrical conductivity. Thus, these two parameters are correlated well in this study. A wider range of EC (473–1406 *μ*Scm^−1^) was reported for drinking water from natural springs in the study area as documented in a previous study [66], which was attributed to differences in geological structures, agricultural activity, and soil conditions within the study area.

The values of TDS are within the range of 36–1063, and the average value is 465 ± 192 ppm. It is obvious that 97.57% of samples are within the acceptable limits of the PSI and the WHO. Only 2.43% of samples have TDS values higher than the PSI acceptable limit, and hence, there are no major concerns regarding the dissolved solids. The TDS is correlated with turbidity: the values of the turbidity are within the range of 0.1–3.63 NTU, and the average value is 0.49 ± 0.76 NTU. All the samples are within the PSI and WHO standards, and hence, there are no concerns regarding the solids. A wider range of turbidity (0.05–9.9  NTU) was reported for drinking water from natural springs as documented in a previous study [66] which was attributed to human activities and an increase in the suspended particulate matter. However, a narrow range of 0–2 was reported for natural springs from other areas (Wadi Al Qilt springs) [74].

The values of the pH are within the range of 6.4–8.12, and the average value is 7.33 ± 0.37. All recorded values satisfy the PSI standards and the WHO [58] guidelines. The water quality in terms of pH is acceptable. These results are close to those reported for drinking water from natural springs [66]. The pH values are related to the total alkalinity. The values of the total alkalinity are within the range of 93.1–354, and the average value is 164 ± 206. This indicates that there are no alkalinity risks from industrial and chemical pollution.

### 3.2. Chemical Parameters

The results of chemical parameters of drinking water in Jenin Governorate along with allowable limits of the PSI [73] standards and the WHO [58] guideline values are presented in Table 6. Table 6 lists the range, the mean, and the standard deviation for each of the following ions: nitrate, nitrite, sulfate, chloride, fluoride, ammonia, sodium, calcium, potassium, and magnesium.

The values of nitrate concentration are within the range of 0–48 ppm, and the average value is 14.52 ± 11.54 ppm. All recorded values satisfy the PSI standards and the WHO [58] guidelines. Similarly, the values of nitrite concentration are within the range of 0–0.86 ppm, and the average value is 0.05 ± 0.03 ppm. All samples satisfy the WHO [58] guidelines. This obtained range for nitrate is narrower than that obtained previously for water from natural springs [66], with some groundwater resources contaminated with nitrate resulting from the penetration of nitrates from sewage and other wastes. However, the obtained range is close to that previously reported for water from springs in other areas (Wadi Al Qilt springs) [74]. Similarly, the values of the ammonia content are in the range of 0–2.63 ppm with an average value of 0.17 ± 0.5 ppm, which is lower than the WHO limit (1.5 ppm). This indicates that there are no risks from ammonia contaminations. Likewise, the values of sulfate concentration are within the range of 1.30–52.94 ppm, and the average value is 22.67 ± 12 ppm. All samples were within the limits of the PSI [73] and WHO [58] guidelines. This indicates that there are no risks from industrial pollution. Similarly, the values of fluoride concentration are within the range of 0.03–3.00 ppm, and the average value is 0.32 ± 0.05 ppm. All the samples are within the limits of the PSI [73] and WHO [58] standards.

Furthermore, the values of chloride concentration are within the range of 113.73–380.05 ppm, and the average value is 96.36 ± 97 ppm. All samples were within the limits of the PSI [73] and WHO [58] guidelines. These results are in line with the results for salinity as presented in Section 3.1 since salinity is correlated with the presence of sodium chloride that releases chloride ions and sodium ions. For a similar correlation, the values of sodium concentration are low, within the range of 9.551–108 ppm, and the average value is 43.42 ± 24.45 ppm. The values of potassium concentration are of ranges between 0.384 and 7.481 ppm, and the average value is 3.00 ± 1.77 ppm. All recorded values of sodium and potassium concentrations are within the limits of the PSI [73] and WHO [58] guidelines, and a previous study [66] indicated that the chloride and sodium contents of water from springs had wider ranges, with some values exceeding the permission limits according to the PSI and WHO.

On the other hand, the values of calcium concentration for 34.6% of the samples are over the PSI standard limits (for samples obtained from wells). The values of calcium concentration are within the range of 1.42–152.90 ppm, and the average value is 78.75 ± 40.20 ppm. The calcium content is dependent on the geological aspects. The contact of water with dolomite and limestone can lead to a high concentration of calcium [75]. High levels of calcium can lead to scaling [76]. These results are correlated with the obtained values of total hardness.  Table 7 shows the water quality classification for various ranges of hardness. Most of the samples are classified as hard or very hard. This leads to the deposition of white scales on the piping systems and may cause kidney stone formation [47].

The results of the contents of heavy metals in drinking water in Jenin Governorate along with allowable limits of the PSI [73] standards and the WHO [58] guideline values are listed in Table 8. Table 8 lists the range, the mean, and the standard deviation for seven types of heavy metals. The concentrations of all heavy metals analyzed (Al, Zn, Fe, Pb, Cr, Ag, and Cu) are below the maximum limits set by the PSI [73] and WHO [58] standards. The concentrations of some heavy metals were found to be below the detection limit of the analytical methods applied. These results indicate that there are no risks associated with heavy metal contaminations.

### 3.3. Microbiological Parameters

Table 9 shows the analytical results of the microbiological parameters in terms of total coliforms, their classifications according to their level of contamination, and the recommended treatment procedure. It is clear that 85.5% of the samples satisfy the acceptable limits of the PSI standard. This means that no treatment is needed for this fraction before using for drinking or cooking. On the other hand, the remaining percentage of the samples (14.5%) is with values exceeding the acceptable limit, and thus, they are contaminated with microbiological pollutants. Among these contaminated cases, 8.71% must use chlorination, 4.4% need flocculation, sedimentation, and chlorination, and 1.71% need advanced treatment using special treatment [12].

Table 10 lists the distribution of tested drinking water samples for fecal coliforms (CFU/100 mL) and their classifications according to their degree of risk. A total of 2494 samples were analyzed for fecal coliforms, 93.30% of these samples possess no risk on health and 2.34% possess moderate risk, 0.9% possess a high risk, and 0.58% possess a very high risk based on the WHO guidelines and classification [12]. The results of total and fecal coliforms indicate that there are sources of microbial pollution, the presence of which is unacceptable for drinking. A previous study [77] indicated that only three communities in Jenin Governorate are connected to the public wastewater collecting system, while 80% of communities use a septic tank for the disposal of wastewater. In areas where there is a high concentration of septic tanks, it is possible for pathogenic organisms to penetrate into wells or nearby surface water [78]. All the polluted samples were taken from the wells and springs.

## 4. Conclusions and Recommendations

The findings of the study show that most of the water quality parameters are within the acceptable limits of the PSI and WHO standards. These include electrical conductivity, turbidity, salinity, pH, total alkalinity, and concentrations of nitrate, nitrite, sulfate, chloride, sodium, potassium, aluminum, and fluoride ions. Furthermore, the concentrations of heavy metals including Zn, Fe, Pb, Cr, Ag, and Cu are within the permission limits, and hence, there is no potential impact on human health. This indicates that there is no impact of industrial pollution or excessive use of fertilizers on water quality within the study area. The findings of the TDS analysis indicate that 97.57% of samples are within the acceptable limits, while only 2.43% are over the limit, which does not affect the human health but can cause the formation of scaling in water pipes, water heaters, and boilers. The findings of the total hardness indicate that the majority of samples are classified as very hard to hard water due to the presence of high amount of dissolved calcium salts. Moreover, 34.61% of calcium samples are over the limit of the PSI.

About 85% of the tested samples for TC show that there is no need for treatment before human use while the remaining percentage of samples are polluted and must be treated for safe use. On the other hand, 93% of the tested samples for FC indicate that there is no risk for human use. Wastewater discharging and unsafe disposal of wastewater are related to the microbial contamination content of TC and FC.

Based on the results of the study, the following recommendations are stated:

- Water treatment for harness removal may be required
- Water disinfection is required for the removal of pathogens
- There is an essential need for the construction of urban sewer systems
- There is a need to increase the number of tests for heavy metals
- There is a need for closing the polluted water sources until treated especially in cases polluted with TC and FC
- There is a need to increase the public awareness of people about the impacts of drinking polluted water

## Figures and Tables

**Table 1:** Water samples for physiochemical and chemical parameters.

Parameter	Number of samples
Conductivity	26
Fluoride (F)	36
Nitrate	42
Nitrite	20
pH	40
Salinity (%)	26
Sulfate (SO_4_)	26
Total dissolved solids (TDS)	41
Total hardness	27
Turbidity	26
Chloride (Cl)	34
Ammonia	30
Calcium (Ca)	26
Magnesium (Mg)	27
Sodium (Na)	26
Potassium (K)	26
Aluminum (Al)	11
Total alkalinity	6

**Table 2:** Water samples for testing heavy metals.

Heavy metal parameter	Number of samples
Ag	19
Cu	19
Zn	19
Fe	19
Pb	19
Cr	19

**Table 3:** Water samples for biological parameters.

Biological parameter	Number of samples
Total coliforms	2570
Fecal coliforms	2568

**Table 4:** Physiochemical parameters of drinking water in Jenin Governorate of the West Bank compared to allowable limits of the PSI standards and the WHO guidelines.

Physiochemical parameter	Range of measured values	Average ± standard deviation	PSI [73] standard limit	WHO [58] limit	Percentage of samples over MCL^a^ of PSI (%)
Conductivity (EC) (*μ*S/cm)	242–1833	890 ± 302	Up to 2000	Up to 2000	0%
Salinity (%)	0.01–0.5	0.1 ± 0.07	NA	NA	NA
Total dissolved solids (TDS) (ppm)	36–1063	465 ± 192	1000	1000	2.43%
Turbidity (NTU)	0.10–3.63	0.49 ± 0.76	5	5	0%
pH	6.40–8.12	7.33 ± 0.37	6.5–8.5	6.5–8.5	0%
Total alkalinity (ppm)	93.11–354	164 ± 206	NA	NA	NA

MCL^a^: maximum concentration limit according to the PSI [73]; NTU: nephelometric turbidity units; ^*∗*^NA: not available.

**Table 5:** Classifications of water quality for various ranges of EC in *μ*S/cm at 25°C.

Range of EC (*μ*S/cm)	Water quality classification [64]	Percentage of samples (%)
<250	Excellent	3.8
250–750	Good	19.2
750–2,000	Permissible	77
2,000–3,000	Doubtful	0
>3,000	Unsuitable	0

**Table 6:** Concentrations of ions in drinking water in Jenin Governorate of the West Bank compared to allowable limits of the PSI standards and the WHO guidelines.

Physiochemical parameter	Range of measured values	Average ± standard deviation	PSI [73] standard limit	WHO [58] limit	Percentage of samples over MCL^a^ of PSI (%)
Nitrate (ppm)	0–48	14.52 ± 11.54	70	50	0%
Nitrite (ppm)	0–0.86	0.05 ± 0.03	NA	3	N.A
Ammonia (ppm)	0–2.63	0.17 ± 0.5	NA	1.5	N.A
Sulfate (SO_4_) (ppm)	1.30–52.94	22.67 ± 12	200	250	0%
Fluoride (F) (ppm)	0.03–3.00	0.32 ± 0.05	1.5	1.5	0%
Chloride (Cl) (ppm)	13.73–380.05	96.36 ± 97	250	250	0%
Sodium (Na) (ppm)	9.551–108	43.42 ± 24.45	200	NA	0%
Potassium (K) (ppm)	0.384–7.481	3.00 ± 1.77	10	NA	0%
Calcium (Ca) (ppm)	1.42–152.90	78.75 ± 40.20	100	NA	34.61%
Magnesium (Mg) (ppb)	0.30–58.33	22.50 ± 15.84	100	NA	0%
Total hardness (ppm)	105.6–549.84	329.42 ± 109.64	500	500	3.7%

MCL^a^: maximum concentration limit according to PSI [73]; ^*∗*^NA: not available.

**Table 7:** Water quality classification for various ranges of hardness.

Total hardness (mg/L as CaCO_3_)	Degree of hardness [63]	Percentage of samples (%)
0–75	Soft	0
75–150	Moderately hard	11
150–300	Hard	15
>300	Very hard	74

**Table 8:** The concentrations of heavy metals in water samples in the study area.

Metal	Average concentration (*μ*g/L)	WHO limit (*μ*g/L)	Palestinian limit (*μ*g/L)	Samples over MCL of PSI (%)
Al	2.79 − 54.13	17.20 ± 16.67	200	0
Zn	20.7 ± 18.2	3000	5000	0
Fe	2.74 ± 2.98	NA	300	0
Pb	0	10	10	0
Cr	0.03 ± 0.091	50	50	0
Ag	0	50	50	0
Cu	6.47 ± 28.21	2000	1000	0

**Table 9:** Distribution of the tested drinking water samples for total coliforms and their classifications according to their level of contamination and the recommended treatment procedure.

Recommended treatment procedure ^*∗*^	Range of total coliforms (CFU/100 mL)	Degree of contamination	Percentage of samples (%)
No treatment	0–3	0	85.53
Chlorination only	4–50	1	8.37
Flocculation, sedimentation, and then chlorination	51–50,000	2	4.40
Very high contamination, needs special treatment	>50,000	3	1.71

^*∗*^[12].

**Table 10:** Distribution of tested drinking water samples for fecal coliforms (CFU/100 mL) and their classifications according to their degree of risk.

Range of fecal coliforms (CFU/100 ml)	Degree of risk^*∗*^	Number and percentage of tested samples (%)
0	No risk	(2396) 93.30
1–10	Low risk	(74) 2.88
11–100	Moderate risk	(60) 2.34
101–1000	High risk	(23) 0.90
>1000	Very high risk	(15) 0.58

^*∗*^[12].

## Data Availability

The data used to support the findings of this study are available from the corresponding author upon request.
